# Children's Motor Intelligence Evaluation System Based on Multi-data Fusion

**DOI:** 10.1155/2022/3775800

**Published:** 2022-09-05

**Authors:** Sihong Zhao

**Affiliations:** School of Preschool Education, Xi'an University, Xi'an 710065, Shaanxi, China

## Abstract

Along with the main feedback information of early childhood education activities, children's movement evaluation plays an important guiding role in early childhood education activities. Teachers can teach children in accordance with their aptitude according to the results of children's sports evaluation. Traditional physical education overemphasizes the leading role of teachers, and young children can only passively receive the education of teachers. Teachers always use the same standard to evaluate each child, simply assigning a rating of “strong,” “moderate,” and “poor” to children, ignoring the differences in children's physical intelligence. The emergence of multidata fusion technology can use the differences and complementarity of various data in evaluation functions to make up for the insufficiency of a single exercise evaluation result, purposefully choose the evaluation method flexibly according to the content of the exercise and the scene of the exercise, and gradually improve the level of children's exercise evaluation. This paper studied the children's motor intelligence evaluation system based on multidata fusion. To this end, this paper will focus on children's autonomous sports games and determine the first-level indicators in the children's sports evaluation index system as four indicators: classroom performance, physical fitness, motor skills, and extracurricular fitness. It used the principle of multidata fusion, firstly evaluates children's exercise physiology data through a fuzzy neural network algorithm, and then combines the adaptive weighted data fusion algorithm with D-S evidence theory to evaluate children's movement intelligence. Experiments showed that the multidata evaluation system can take effective measures to intelligently evaluate children's comprehensive motor ability. Compared with the traditional evaluation method, the evaluation results are increased by 5%, and the children's sports evaluation results are more average, which can enhance children's sports confidence and promote children's effective exercise.

## 1. Introduction

The perspectives of children's sports evaluation are becoming increasingly diversified. In the past ten years, many theoretical and practical workers in China have tried to explore the strategies and methods of children's sports evaluation from various perspectives, mainly introducing foreign evaluation theories and discussing the reference significance of this theory to China's children's sports evaluation. Therefore far, different tools have been used abroad to evaluate young children's motor ability. Exercise assessment tests can be standard references or normative references. At present, the research on children's movement evaluation under the background of multidata fusion in China is only in its infancy, and a scientific evaluation system has not been formed. A single sports evaluation cannot tap children's sports potential. To respect children's differences and stimulate their creative potential, it is necessary to establish a multidata children's sports evaluation system with multiple integration and flexible evaluation. The normative reference test compares the performance of the average child to a normative sample population and quantifies the ability of children to motor skills. Standard reference tests compare children's abilities with predetermined standards. Standard reference tests take into account the qualitative aspects of motor skills required to perform in sports and are mainly evaluated by teachers through testing scales for minors. At present, many scholars have carried out research on children's movements, and the research includes many aspects. Francesca et al. investigated questions about core sports values between parents and children through questionnaires. The survey results showed that young athletes are generally willing to accept their parents' socialized values in sports [1]. Using semistructured interviews, Watchman and Spencer-Cavaliere examined parents' perceptions of children's free play and movement from a socioecological perspective, capturing how children's movement and free play have evolved since their parents' childhood. The conclusions demonstrate that freedom of play and physical activity are considered important for midchildhood, whereas the experience gained in children's physical activity is considered more valuable for the overall development of the child [2]. McGowan et al. investigated the relationship between early specialization and sports participation and injury history in New Zealand children through questionnaires, and the probability of reporting injury history in early professional children was not significantly higher than that of low professional children [3]. The results of Costi et al.' questionnaire study describing the distribution of scores on the Activity Performance Scale for Children (ASKP) in an Italian school-age population offer the first proof of the validity of the Italian version of the ASKP construct which will help clinicians to interpret ASKP scores in children with musculoskeletal limitations [4]. Sirard and Pate found 59 articles validating physical activity measures in children and adolescents through MEDLINE searches and journal article citations, summarizing the strengths and limitations of methods used to assess physical activity in children and adolescents [5]. Gorman et al. studied the principles of children's sports equipment upgrade methods through basketball case studies. This research aims to illustrate how a principled approach to hand anthropometry can be used to determine the optimal basketball size for youth basketball players by measuring hand width and length in youth and older male basketball players and used to create hand size-to-ball ratios [6]. Howard et al. investigated whether early childhood (age 4-5) participation in physical activity predicts changes in children's selfregulation two years later. The results showed that toddlers who participated in individual sports exhibited higher selfregulation abilities than those who did not [7]. Although there are many studies related to child evaluation, the current research is less related to the research on child movement evaluation system, and the type of movement evaluation data is relatively simple.

The multidata fusion research method can solve the problem of a single data type and has been widely used in various fields. Yan et al. introduced a method to simulate EHR composed of multiple data types. An analysis of more than 770,000 electronic medical records showed that the new model achieved higher performance in preserving basic statistics, cross-feature correlations, underlying structural properties, feature constraints, and association patterns in real data, while not sacrificing privacy [8]. Rahimi et al. collected and identified 18 species of Plasmodium from different regions and defined these species based on multiple datasets and by using bioinformatics and phylogenetic methods. Studies have shown that the task of phylogenetic and phylogenetic studies requires comprehensive data analysis of pili species [9]. Ghosh et al. utilized a variety of data sources corroborated by comprehensive field inspection. They compiled a largely complete landslide inventory of landslide numbers and attributes to understand the role of landslide behavior and triggers in sensitivity mapping, as well as the geological and environmental conditions that determine the event scales [10]. Huang et al. used 3 data-driven models to simulate and predict the monthly runoff series at the hydrological station from 1981 to 2017, to improve accuracy and reduce uncertainty. Applying two model averaging techniques to combine the prediction results of different models, it was found that the random forest (RF) algorithm has almost the same accuracy as the artificial neural network algorithm [11]. Verma et al. presented a QOS-provisioned routing protocol that uses multiple data sinks in WSN-based IoT to mitigate the hotspot problem by circumventing multihop communication. Their performance has been evaluated based on the performance metrics provided by QOS, and the simulation results obtained confirm that the proposed protocol outperforms the state-of-the-art protocols [12]. In developing a flounder classifier for systematic fish management in aquaculture, Hwang et al. considered a multisensor data fusion system using load cells and vision sensors to compensate for motion disturbances. He evaluated the performance of the algorithm by comparing single-sensor measurements and multisensor data fusion results [13]. Li and Gan built a multisource data fusion model based on an ensemble learning algorithm. The results show that, according to the results of multisource tourism information fusion, the model prediction accuracy after data processing is about 62% [14]. At present, there are few research studies on multidata fusion in children's movement evaluation system. To study a more flexible and intelligent evaluation system, this paper introduces multidata fusion into children's movement evaluation.

On the basis of fully analyzing the characteristics of children's sports data, this paper determines the first-level indicators in the children's sports evaluation index system as four indicators: learning attitude, physical fitness, team sports skills, and extracurricular fitness. The weight of each first-level index in the evaluation of children's movement is 0.1, 0.5, 0.2, and 0.2, respectively. It uses the method of multidata fusion analysis, firstly evaluates children's exercise physiological data through fuzzy neural network algorithm, then uses SPSS software based on the D-S evidence theory algorithm for statistical processing of data, and obtains the results of children's movement evaluation. 60 children in a kindergarten were selected as experimental objects and divided into an experimental group and a control group, each group including 10 students in a small class, a middle class, and a large class. Afterwards, the children's movement experiment was carried out to study the scientific multidata fusion children's movement evaluation system.

The innovation of this paper is as follows:

1. Preliminary evaluation of children's exercise physiology data through fuzzy neural network algorithm
2. It uses the adaptive weighted data fusion algorithm for data fusion
3. It uses the D-S evidence theory algorithm to evaluate the movement of young children

## 2. Structure of the Multidata Fusion Children's Movement Evaluation System

This paper proposes a multi-data fusion evaluation of children's movement. After classifying and merging the multi-index data, the children's movement is intelligently analyzed according to the weight of each index. The functional model of data fusion starts from the fusion process and describes the main functions, databases, and the interaction process between the various components of the system during data fusion [15]. The functional model of data fusion can be divided into five layers, namely, primary detection fusion, second-level location fusion, third-level attribute target recognition fusion, fourth-level processing, and fifth-level processing. The functions cover detection, judgment, prefiltering, acquisition, management, tracking, classification, evaluation and reasoning, threat estimation, database management, support database, situation database, human-machine interface, and performance evaluation. The functional model of data fusion is shown in Figure 1.

### 2.1. Exercise Evaluation Based on Fusion of Physiological Data

#### 2.1.1. Physiological Data Fusion Model

Functionally, the physiological data fusion model includes the acquisition of multisource heterogeneous physiological sensor information, data calibration, filtering and association merging of the second-level location and state fusion, third-level attribute fusion, and the fourth-level situation assessment. The multisensor acquisition part is composed of a series of multisource heterogeneous and high real-time physiological sensors. The main function is to collect the physiological index data of the dynamic changes of the human body in a certain process as a fusion information source [16]. The schematic diagram of sensor information acquisition is shown in Figure 2.

It can be seen from Figure 2 that when the sensor set collects information, the information is first collected through the sensor nodes, and then the information is transmitted to the gateway node, and the gateway node transmits the information to the control center through the sensor network.

### 2.2. Physiological Data Fusion Model Algorithm Research

Neural network has strong advantages in learning and automatic pattern recognition. Fuzzy neural network is the introduction of fuzzy logic in neural network, which enables it to directly process fuzzy information [17]. It has various structural forms, one of which is a simple form of fuzzification and defuzzification at the input and output layers of the neural network, respectively.

#### 2.2.1. Motion Evaluation Based on Adaptive Weighting Algorithm and D-S Evidence Theory

After each motion index data is fused according to a weighting algorithm, motion evaluation is performed according to the D-S evidence theory. The scheme of the data fusion evaluation system is shown in Figure 3.

### 2.3. Data Analysis and Decision-Making Based on D-S Evidence Theory

Evidence theory is a mathematical theory of evidence-based reasoning that deals with problems that lead to uncertainty due to ignorance [18]. It can combine different types of interrelated evidence to achieve the purpose of fusion analysis of a variety of different evidence to reach the final conclusion. The data analysis and decision-making structure is shown in Figure 4.

## 3. Multidata Fusion Child Movement Evaluation System Algorithm

### 3.1. Physiological Data Fusion Model Algorithm

The first layer is the fuzzification layer, which is mainly to quantify the input data of human physiological indicators and realize the fuzzification of the true value information through the membership function. The input vector *I*1 corresponds to the feature value *S*_out_ of each physiological sensor, after primary fusion processing, the node transfer function corresponds to the relevant membership function, and the output feature value *O*1 is the membership function value corresponding to each fuzzy set. The semantic quantifiers describing human physiological indicators are determined as high (fast), normal, and low (slow), and the types and parameters of each membership function are determined according to the distribution characteristics of human physiological indicator signals.

(1) $$\begin{array}{c} I1=S_{\text{out}},\\ O1=\mu \left(I1\right). \end{array}$$

Among them, *μ* is the membership function of the input vector *I*1.

The second layer is the quantized input layer, which corresponds to the input of the general BP network. The membership function output by the first layer node is used as input, and the node transfer function is selected as tansig.

(2) $$\begin{array}{c} I2=O1,\\ O_{2}=\text{tansig}\left(I2\right)=.\frac{2}{1+\text{exp}\left(-2\times I2\right)}-1. \end{array}$$

The third layer is the hidden layer of the fuzzy neural network, which is similar to the hidden layer of the network. Using the learning of typical sample data, through the continuous correction and adjustment of weights and thresholds, the mapping relationship between the input physiological information and the fusion target output is established, and the transfer function is a logarithmic function.

(3) $$\begin{array}{c} I_{3j}=\sum_{i=1}^{m}\left(w_{ij}o_{2i}-\theta_{j}\right),\\ O3=\text{logsig}\left(I3\right)=\frac{1}{1+\text{exp}\left(-I3\right)}. \end{array}$$

The fourth layer is the quantized output, which is equivalent to the output layer of the BP neural network, and the node transfer function is tansig.

(4) $$\begin{array}{c} I4=\sum_{j=1}^{n}\left(w_{j}o_{3}-\theta_{k}\right),\\ O4=\text{tansig}\left(I4\right)=\frac{2}{1+\text{exp}\left(-2\times I4\right)}-1. \end{array}$$

The fifth layer is the defuzzification layer, which mainly defuzzifies the output value of the fourth layer. The fuzzy quantized value is converted into a true value output through the inverse solution of the membership function.

### 3.2. Data Analysis and Decision-Making Based on D-S Evidence Theory

Evidence theory data fusion rules are as follows [19, 20]:

If *m*_1_(*A*) and *m*_2_(*A*)(*A* ∈ 2^*U*^) are the two basic probability distribution functions of *U* based on different evidence, then after combining according to the combination rules of evidence theory:

(5) $$\begin{array}{c} m\left(A\right)=\left\{\begin{array}{cc} 0 & A=\Phi \\ K\sum_{N\cap C=A}m_{1}\left(B\right)m_{2}\left(C\right) & A\neq \varphi \end{array}\right., \end{array}$$

where

(6) $$\begin{array}{c} K={\left(1-\sum_{B\cap C=A}m_{1}\left(B\right)m_{2}\left(C\right)\right)}^{-1}. \end{array}$$

*m*(*A*) is the orthogonal sum of all probability assignment functions.

Evidence theory has a strong theoretical foundation. Through the accumulation of evidence, the hypothesis set can be continuously reduced. The complexity of time and information is low, and it has a good effect in dealing with uncertain problems caused by ambiguity.

## 4. Experimental Children's Movement Evaluation

### 4.1. Experimental Object

60 children in a kindergarten were selected as experimental subjects, 30 of whom were the experimental group and 30 were the control group.

### 4.2. Experimental Method

In the control group, children were evaluated using traditional evaluation criteria. The experimental group determined four evaluation indicators, namely, learning attitude, physical quality, teamwork ability, and extracurricular sports. The weights of each first-level index in the children's sports evaluation were 0.1, 0.5, 0.2, and 0.2, respectively. This paper uses the method of multidata fusion analysis to evaluate children's motor intelligence. The evaluation results of the two groups were compared, and the differences and advantages and disadvantages of the two evaluation methods were analyzed.

#### 4.2.1. Observation Method

Teachers observe the interaction of children in sports activities under the state of natural observation and use cameras to shoot the whole process to objectively evaluate children's learning attitudes and team sports skills. The evaluation grades are divided into good, good, general, poor, and poor. Each grade is scored as 10, 8, 6, 4, and 2, and the average score of the five teachers' evaluations is taken as the final score.

#### 4.2.2. Measurement Method

After reading a lot of literature on children's sports, seven items, 20-meter running, standing long jump, sandbag, throwing, ball sling, single-leg jumping, and double-arm support, were selected as the physical fitness measurement and evaluation indicators for children. According to different classes and genders, it uses fuzzy neural network algorithm, 10%, 25%, 50%, 75%, and 90% quantile method, grading, and fusion of various sports data, and the scoring interval is 1-10 points.

#### 4.2.3. Interview Method

The parents of young children were interviewed about their children's extracurricular sports abilities. The interviews included children's extracurricular sports items, the length of extracurricular sports, and the initiative of children's extracurricular sports, and the children's extracurricular sports ability was objectively rated. The evaluation grades are divided into good, good, fair, poor, and poor, and each grade is scored as 10, 8, 6, 4, and 2. The average score of 5 teachers' evaluations was taken as the final score.

#### 4.2.4. Mathematical Statistics

The first-level indicators in the children's sports evaluation index system are determined as four indicators: learning attitude, physical fitness, team sports skills, and extracurricular fitness, and the weights of each first-level index in the children's sports evaluation are 0.1, 0.5, 0.2, and 0.2. According to the adaptive weighted data fusion algorithm and the D-S evidence theory algorithm, the collected data is statistically processed by SPSS social statistical analysis software, and a scientific evaluation of children's motor intelligence is given.

## 5. Data of Children's Movement Evaluation Experiment

### 5.1. Evaluation of Learning Attitude in the Experimental Group

In this experiment, 5 teachers were selected to observe children's learning attitude, individual motor skills, and team motor skills during daily exercise and objectively score each child. After removing the highest score and the lowest score, the remaining results are averaged, which is the final score of the indicator. The results of classroom performance and motor skills evaluation of the experimental group are shown in Figure 5.

Taking 6 points as the pass line, it can be seen from the data in Figure 5 that the pass rate of students in the big class is 80%, the pass rate of students in the middle class is 80%, and the pass rate of students in the small class is 90%. There is no significant difference in the data of the three classes, indicating that more than 80% of the children have a serious learning attitude and a greater interest in sports. When conducting a comprehensive evaluation of athletic ability, the learning attitude of most children has little effect on the final result, and students with higher or lower learning attitudes will have a higher or lower overall score on this indicator.

### 5.2. Evaluation of Team Sports Skills in the Experimental Group

5 teachers were selected to observe children's team sports skills during their daily movements and objectively score each child. After removing the highest score and the lowest score, the remaining results are averaged, which is the final score of the indicator. The results of the team sports skill evaluation of the experimental group are shown in Figure 6.

As for the teamwork ability of young children, it can be seen from the data in Figure 6, that the ability of students in the three classes to unite and cooperate in descending order is the large class, the middle class. and the small class. Pass rate of teamwork among large class students is 90%, and three of them have a teamwork ability of more than 8 points, and one of them has a score of 9 points or more. The teamwork pass rate of middle class students is 80%, and the teamwork ability of the three students reached 8 points. The teamwork pass rate of the small class students is 80%, and there are two students whose teamwork ability is above 8 points. Comparing the data of the three classes, it can be seen that the overall teamwork ability and awareness of the students in the large class are better than those in the middle class and the small class, indicating that with the growth of age, the children's teamwork ability has improved, and they gradually realize the importance of teamwork.

### 5.3. Evaluation of Extracurricular Sports Ability of the Experimental Group

Five teachers were selected to conduct interviews with parents of young children about their children's extracurricular sports abilities. Next, objectively score each child, remove the highest score and the lowest score, and take the average of the remaining results, which is the final score of the indicator. The results of the extracurricular sports ability evaluation of the experimental group are shown in Figure 7.

Regarding the extracurricular sports ability of young children, it can be seen from the data in Figure 7 that the pass rate of extracurricular sports ability of large class students is 70%, and two of them have achieved extracurricular sports ability of 8 points or more. In the middle class, 80% of the students also reached the pass line or above, and three of them achieved excellent extracurricular sports ability, one of whom achieved a score of 9 or more. 80% of the students in the primary class reached the pass line, and two of them achieved 9 points, and the overall extracurricular sports scores were relatively high. Comparing the data of the three classes, it can be seen that the children's overall extracurricular athletic ability is in the small class, middle class, and the large class in descending order, indicating that the younger children have greater enthusiasm for sports. Taking extracurricular sports as one of the sports evaluation indicators can encourage children to exercise autonomously in daily life and improve their enthusiasm for sports.

### 5.4. Physical Fitness Evaluation of the Experimental Group and the Control Group

Seven items including 20-meter running, standing, long jump, sandbag throwing, ball smashing, single-leg jumping, and double-arm support were selected as the measurement and evaluation indicators of children's physical fitness. Both groups of children were tested for physical fitness, and the fuzzy neural network algorithm was used for data evaluation. The physical fitness results of the experimental group are shown in Figure 8, and the physical fitness results of the control group are shown in Figure 9.

For the physical fitness data of the experimental group, it can be seen from Figure 8 that 70%, 80%, and 80% of the students in the large class, the middle class, and the small class achieved a score of 6 or above, respectively, and the excellent rate of each class was 40%, 40%, and 30%. Among them, one person in the large class achieved a score of 9. For the data of the control group, it can be seen from Figure 9 that 80%, 70%, and 80% of the students in the large class, the middle class, and the small class, respectively, reached the passing grade, and the excellent rate of each class was 30%, and a total of 3 students achieved 9 points. Comparing the data of the experimental group and the control group, it is found that the overall difference is small, and more than 70% of the children have good physical fitness, indicating that the physical fitness of the two groups of subjects in this experiment is similar, and the difference in physical fitness has little impact on the final comprehensive evaluation of athletic ability.

### 5.5. Comprehensive Evaluation of the Exercise Ability of the Experimental Group

For the experimental group, the above sports index data were fused according to the weight, and the SPSS analysis software was used for statistical processing to obtain the results of children's sports evaluation. The exercise evaluation results of the control group are the physical fitness evaluation results, and the results of the two groups are compared and analyzed. The exercise evaluation results of the experimental group are shown in Figure 10.

As can be seen from Figure 10, after the weighted and integrated evaluation of various index data, the pass rate of the experimental group's athletic ability is 90% in the large class, 80% in the middle class, and 80% in the small class. The overall data is relatively average. Comparing Figure 10 with Figures 8 and 9, it can be seen that after the four indicators of learning attitude, physical quality, team sports skills, and extracurricular fitness are integrated and evaluated, the overall sports ability evaluation of children has improved, and the data lines have become smoother, compared with the single-motion evaluation results, the data is improved by 5%. It shows that children's positive learning attitude and good teamwork can improve the overall sports evaluation, and the evaluation results are more comprehensive and reasonable.

## 6. Experiment Results and Discussion of Children's Movement Evaluation

The traditional sports evaluation of children takes the physical quality of children as the only standard, ignoring the differences and development potential of children in sports intelligence. The introduction of multidata fusion technology into children's movement evaluation can make up for the shortcomings of a single evaluation method and conduct targeted and flexible evaluations according to different children. In this paper, multidata fusion technology is integrated into children's sports evaluation, and a more intelligent sports evaluation system is studied.

1. This paper selected 7 items of 20-meter running, standing, long jump, sandbag throwing, batting on the spot, single-leg jumping, and double-arm support as the measurement and evaluation indicators of children's physical fitness. It conducted a preliminary evaluation on children's exercise physiology data through fuzzy neural network algorithm and compared the data between the experimental group and the control group. The experimental results showed that the physical fitness of the two groups of subjects in this experiment is similar, and the difference in physical fitness has little effect on the comprehensive evaluation of the final exercise ability.
2. This paper determined the evaluation index in the children's movement evaluation index system, collected the data of each index of children, and fused the data of each index according to the adaptive weighted data fusion algorithm. The adaptive weighted data fusion algorithm can perform data fusion according to the weight of each index, and the algorithm is more intelligent and reasonable.
3. Based on the D-S evidence theory algorithm, this paper used the social statistical analysis software SPSS to statistically process the collected data and compared the comprehensive exercise evaluation data of the experimental group with the single physical fitness data of the control group. It can be seen that, compared with the single evaluation results, after the fusion of various index data, the children's evaluation results are more average. Also, the overall evaluation results have improved. Children with moderate physical fitness data can also improve their sports evaluation results through learning attitudes, teamwork ability, and extracurricular sports abilities, which can enhance children's sports confidence and enhance children's sports enthusiasm.

## 7. Conclusion

This paper collects four movement index data of children and uses the method of multidata fusion analysis. It first evaluates children's movement physiological data through fuzzy neural network algorithm, then uses the idea of adaptive weighted data fusion algorithm for data fusion, and uses the D-S evidence theory algorithm to evaluate children's movement. The experimental results show that after the fusion of various index data, the evaluation results of children are more average, and the overall evaluation results are improved. The multidata fusion evaluation system can evaluate children's comprehensive sports ability in an all-round way, and the evaluation results are improved by 5% compared with the traditional evaluation method.

## Figures and Tables

**Figure 1:** Data fusion functional model.

**Figure 2:** Schematic diagram of sensor information collection.

**Figure 3:** Data fusion evaluation system scheme.

**Figure 4:** Data analysis and decision-making structure diagram.

**Figure 5:** Evaluation chart of the learning attitude of the experimental group.

**Figure 6:** Evaluation of team sports skills in the experimental group.

**Figure 7:** Evaluation chart of the extracurricular sports ability of the experimental group.

**Figure 8:** Physical fitness evaluation chart of the experimental group.

**Figure 9:** Physical fitness evaluation chart of the control group.

**Figure 10:** Comprehensive evaluation table of exercise ability of the experimental group.

## Data Availability

Data sharing not applicable to this article as no datasets were generated or analyzed during the current study.
